# Analysis of Marine Economic Development and Innovation under Environment Constraint Based on the VAR Model

**DOI:** 10.1155/2022/5392014

**Published:** 2022-07-13

**Authors:** Danjie Wu

**Affiliations:** Fujian Jiangxia University, Fuzhou 350108, China

## Abstract

Building a new development pattern based on the “double-cycle” is a major strategic plan of China. Under the background of the new development pattern of the “double-cycle” and the context of environmental constraints, this paper tries to explore the impact of marine economic development on marine cultural industry and marine innovation development, the extent of the impact of marine cultural industry on marine economic growth, and the internal relationship between them under the new development pattern of double circulation. In this paper, Fujian Province is taken as the research object to construct an indicator system of the marine culture development to reflect the living standard, employment level, and spiritual and cultural levels of people in the marine area, and the external influence of the marine economy and marine culture industry is taken as the indicator variable to measure the integrated development. The internal changes are regarded as the index to assess the integration level of the two, and the evaluation theoretical model of the dynamic evolution level of the marine economy and marine cultural industry is constructed. The vector autoregression model and impulse response function are used to study the interactive correlation between the growth of the marine economy and the development of the cultural industry. The results show the following: In the long run, there is a cointegration relationship between the marine culture industry and the gross ocean product (GOP), which is a long-term balanced and stable relationship. The development level of the marine economy and the development of marine culture industry are mutually influencing and promoting.

## 1. Introduction

China's gross marine product increased from 6,969.4 billion yuan in 2016 to 8001 billion yuan in 2020. Except for coastal tourism, the marine industry has recovered rapidly and steadily, its scale has continued to expand, and the added value of the industry has bucked the trend. The report to the 19th CPC National Congress said China's economy has shifted to a stage of high-quality development and must adhere to the “five development concepts” and the goal of building a maritime power. The outline of the 14th Five-year Plan, which will be issued in March 2021, clearly states that important plans will be made for the development of marine undertakings from a strategic perspective, and calls for building China into a maritime power and expanding the space for the development of the marine economy. In 2015, the State Oceanic Administration designated the “West Coast of the Straits” as one of China's five marine cultural circles. “Fujian on the Sea” is China's first local documentary on marine topics, and fully demonstrates resource endowment and distinctive cultural deposits of “Fujian on the Sea.” “Fujian Volume of Chinese Marine Culture” calls Fujian traditional shipbuilding and navigation technology “The fifth great invention of China,” and calls Fujian people “the most marine ethnic group in China” and praises Fujian maritime merchants as “no empire.” Fujian marine culture has a top position in the history of Chinese marine culture. During the 13th Five-Year Plan period, Fujian province also proposed that Fujian province should accelerate the construction of emerging industries such as the marine culture industry, coastal tourism, marine sports, leisure industry, sea-related financial service industry, and constantly improve the competitiveness of the marine economy. In 2021, the action plan of “Fujian On the Sea” will promote the marine culture industry to become a “sunrise industry.” In this context, this paper tries to explore the impact of marine economic development on marine cultural industry, the extent of impact of marine cultural industry on marine economic growth, and the internal relationship between them under the new development pattern of double circulation. The answers to these questions will provide a theoretical basis for the government to formulate effective policies and have a practical significance for the high-quality development of the marine economy.

## 2. Literature Review

American economist Gerald J. Mangon (1982) first proposed the concept of “marine economy” in American Ocean Policy. Charles believes that “marine economy is an economic activity that takes marine resources as an input” [1]. Some scholar believes that “marine economy refers to economic activities that provide products and services, and part of the value of these products and services is determined by the ocean or its resources.” This paper analyzes the current situation of the development of the marine economy in the United States and puts forward some countermeasures. Rochwulaningsih et al. by listing examples of the rapid development of marine economy in Indonesia through the dissemination of marine culture and maritime trade in history, believe that the Indonesian government should rebuild marine culture and formulate a comprehensive marine economy development strategy to reflect prominent marine characteristics [2]. From the perspective of the ecosystem, Winther et al. proposed the IOM method to integrate and balance different marine uses, optimize the marine economy as a whole, and achieve sustainable development [3]. Lubchenco et al. proposed five countermeasures to promote the sustainable development of the marine economy from the perspectives of climate change, marine fishing, and biodiversity [4]. China began to study the marine economy in the 1980s. Although it was much later than foreign countries, after years of exploration and development, domestic scholars have also conducted a large number of studies on the marine economy and marine culture from various perspectives. Solow internalized labor productivity and initiated the study of long-term economic growth from the perspective of supply [5]. Subsequently, Lucas internalized human capital [6], Romer [7], and Grossman et al. internalized technological progress as the source of economic growth [8–10]. Furthermore, Nadiri found that technological progress is the result of enterprise R&D, which can explain almost half of the total factor productivity growth [11]. Based on this, some scholars also considered the influence of knowledge spillover effect on economic growth. Different from previous studies, Acemoglu no longer regarded technological progress as endogenous [11], and proposed a technology-biased endogenous economic growth model based on the Dixit-Stiglitz model (Dixit et al.), which has been widely promoted [12]. Biased technological progress means that if the output change brought by the input of the factor is greater than the change of the input [13–15], then the technology progress is biased to the factor [16]. In reality, technology progress is usually biased. With the deterioration of the global environment, more and more scholars consider the impact of resources and the environment on economic growth. With the development of China's marine economy, the pressure on the marine ecological environment gradually increases [17]. From the perspective of research objects, existing scholars' studies mainly include marine fisheries [17] and port technical efficiency [18]. Levinsohn-Petrin (LP) method is adopted by mathematicians to study marine economic efficiency. In the field of the marine economy, based on the super-efficiency DEA (SE-SBM) and the Generalized Method of Moments (GMM) model, Zheng et al. found that in a certain period, Capital input and scientific and technological innovation have a negative effect on marine economic efficiency [19].

Based on the above literature research, it can be seen that as a new industry combining marine economy and culture, the marine cultural industry has a promising development prospect. Existing literature confirms that the marine culture and marine economy can influence each other, and most scholars analyze them from the perspective of marine culture and marine economy. However, few studies focus on the marine cultural industry, especially the lack of empirical analysis on the internal correlation between the marine culture industry and the marine economy. In view of this, drawing on previous experience, this paper aims to deeply analyze the long-term dynamic equilibrium relationship between the growth of the marine economy and the development of the marine culture industry in Fujian Province. Through the stability test and cointegration test of variables, the vector autoregressive model is constructed to test the endogenous interaction relationship between the marine culture industry and the development of the marine economy.

## 3. Empirical Analysis

### 3.1. Variable Selection

To objectively and comprehensively measure the marine economy and marine culture industry development level, fully consider the development of Fujian coastal areas, from the Marine industry development level, export trade development level, and infrastructure development level three dimensions to describe the development of marine economy, choose gross ocean product (GOP) represents marine industry development level, import and export total (MEV) represents import and export trade development level, total fixed assets investment (FAI) represents infrastructure development level. From the marine area, people's living standards, people's employment level, people's spiritual culture level three dimensions to depict marine culture industry development level, urban residents' disposable income level (UPDI) on behalf of marine area people's living standards, the third industry employees (TIE) on behalf of marine people's employment level, books published (BP) represents the marine area people's spiritual culture level. To sum up, the specific descriptions of the marine economy and marine culture industry development index variables are shown in Table 1.

### 3.2. Data Sources

The data of all indicators are from Fujian Statistical Yearbook, China Marine Statistical Yearbook, China Marine Economic Development Report, etc. The detailed original data are shown in Table 2.

### 3.3. Empirical Research on the Relationship between Marine Cultural Industry and Marine Economy Based on Pillar Industry Indicators

#### 3.3.1. Proportion of Marine Cultural Industry in Gross Marine Product

Generally speaking, the industry that accounts for a significant proportion of the economic aggregate in a certain field will have an impact on the economic development of the field. To facilitate comparison, this paper lists the proportion of the marine culture industry, maritime transportation industry, and marine fishery in the total marine GDP from 2010 to 2021, as shown in Table 2. Different from the continuous decline of marine traffic and fisheries, the marine culture industry has an overall growth trend and will account for about 1/5 of the gross marine product by 2021, exceeding the requirement of 5% as a pillar.

#### 3.3.2. Elasticity of Income Demand of China's Marine Culture Industry

The elasticity of demand income refers to the ratio of the increase rate of demand for a certain industrial product to the increase rate of per capita national income. If the elasticity of demand income is greater than 1, it indicates that within the increase of income, demand grows faster than income. Obviously, with the growth of per capita national income, selecting industries with high elasticity of demand income conforms to the law of the market, which is conducive to the evolution of industrial structure and has a great impact on the economy. Since there is no concept of per capita GROSS marine Product, this paper selects the increase of the Marine cultural industry and per capita GROSS Marine product from 2010 to 2021 to calculate the elasticity of demand income. The data in Table 3 were obtained through formula calculation.

#### 3.3.3. Elasticity Analysis of Sea-Related Employment

Elasticity of employment refers to the rate of employment growth caused by each additional unit of the economy under the condition that other factors remain unchanged. If the elasticity of employment is greater than 1, it indicates that the employment capacity brought by economic growth is large and the development of this industry can drive employment and stimulate economic growth. This paper selects the statistical data of marine-related employment from 2015 to 2020 and the added value of the marine cultural industry as the basis for calculating the elasticity of employment. According to the data in Table 4 obtained through formula calculation, although China's marine cultural industry continues to grow, the elasticity of sea-related employment in China is far less than 1, which means that the increase in China's marine cultural industry cannot drive the increase of sea-related employment.

### 3.4. ADF Unit Root Test

ADF (Augmented Dickey-Fuller) test can be used to test the stationarity of time series. If it is not stable, it is necessary to eliminate the unit root by difference, so that the time series can reach the same order integration, and then continue the subsequent tests. The unit root test ADF method was used to conduct unit root test on gross ocean product (GOP), total import and export (MEV), total fixed investment (FAI), urban residents' disposable income level (UPDI), number of tertiary industry employees (TIE) and total books published (BP). The specific test results are shown in Table 5.

As can be seen from the unit root test results in Table 6, the original time series of gross ocean product (GOP), total import and export volume (MEV), urban residents' disposable income level (UPDI) and total books published (BP) are all unstable. After the first-order difference, gross ocean product (GOP) and total fixed investment (FAI) are still unstable. All other variables are stationary. After the second-order difference between gross ocean product (GOP) and total fixed investment (FAI), other variables except for total import and export (MEV) and total fixed investment (FAI) are in a stable state. Here, total import and export (MEV) and total fixed investment (FAI) are excluded, and gross ocean product (GOP) is simplified to represent the development level of the marine economy.

### 3.5. Co-Integration Test

Taking gross ocean product (GOP) as an explanatory variable, urban residents' disposable income level (UPDI), number of tertiary industry employees (TIE), and the total number of books published (BP) as explanatory variables, a cointegration test was conducted. The residual sequence equation and cointegration test results are shown in Tables 7 and 8.

As can be seen from Table 5, there is a cointegration relationship between the number of tertiary industry employees (TIE) and the total number of books published (BP), and there is a long-term correlation between GOP, TIE, and BP. Granger causality test can be continued, to further explore the causal relationship between these endogenous variables.

### 3.6. Granger Causality Test

The stability of the VAR model should be checked before the Granger causality test to avoid false regression.

(1) $$\begin{array}{c} y_{i}=\sum_{i-1}^{q}\alpha_{i}x_{t-i}+\sum_{j-1}^{q}\beta_{j}y_{t-j}+u_{1t}^{4}, \end{array}$$

(2) $$\begin{array}{c} x_{i}=\sum_{i-1}^{s}\lambda_{i}x_{t-i}+\sum_{j-1}^{s}\delta_{j}y_{t-j}+u_{2t}^{4}. \end{array}$$

From the above formula, we can judge the relationship between *x* and *y* in the Granger causality test. Before the Granger causality test, VAR modeling should be carried out. The modeling data of the VAR model are shown in Table 9.

It can be evaluated from Table 10 that the VAR selects 4-order lag order. The significance level of the Granger causality test is set as 10%. When the *P* value of the Granger causality test is less than the significance level, it is proved that the explanatory variable is the Granger Number of the explained variable. The results of the Granger causality test are shown in Tables 11 and 12.

It can be found from Tables 11 and 12 that, firstly, when the explained variable is gross ocean product (GOP), urban residents' disposable income level (UPDI) is the Granger cause of GOP; The number of tertiary industry employees (TIE) and the total number of books published (BP) is not the Granger reason for the gross ocean product (GOP). Secondly, when the explained variable is urban residents' disposable income level (UPDI), gross ocean product (GOP) is the Granger cause of urban residents' disposable income level (UPDI). Thirdly, when the explained variable is the number of tertiary industry employees (TIE), gross ocean product (GOP) is also the Granger cause of the number of tertiary industry employees (TIE). Fourthly, when the explanatory variable is the total number of books published (BP), the gross ocean product (GOP) is the Granger cause of the total number of books published (BP). To sum up, the development level of the marine economy is the Granger cause of the development of the marine culture industry, but the development level of the marine culture industry is not the Granger cause of the development of the marine economy.

### 3.7. Stability Test

Only when the VAR model is stationary, the impulse response convergent, and the analysis is of economic significance. Therefore, the stationarity test of the established VAR model should be carried out. The value of the characteristic polynomial determines the stability of the VAR model. As the lag length of the model is 2 and there are 4 endogenous variables, the unit root of this model has 2 × 4 unit-roots. In this paper, the established VAR model is stable with a test.

## 4. Conclusions and Suggestions

Building a new development pattern based on the “double-cycle” is a major strategic plan of China. Fujian province has rich and profound marine cultural resources and deposits. How to enhance the driving force of marine culture in marine economic growth is not only the inevitable requirement for Fujian province to respond to and integrate into the national strategic deployment and build a new development pattern, but also the only way to meet people's demands for high-quality culture and a better life. Under the background of the new development pattern of the “double cycle,” Fujian Province is taken as the research object to construct an indicator system of marine culture development to reflect the living standard, employment level and spiritual and cultural level of people in the marine area, and the external influence of marine economy and marine culture industry is taken as the indicator variable to measure the integrated development. The internal changes are regarded as the index to evaluate the integration level of the two, and the evaluation theoretical model of the dynamic evolution level of marine economy and marine cultural industry is constructed. The vector autoregression model and impulse response function are used to study the interactive correlation between the growth of marine economy and the development of cultural industry. The results show that: In the long run, there is a co-integration relationship between the marine culture industry and the gross ocean product (GOP), which is a long-term balanced and stable relationship. The development level of marine economy and the development of marine culture industry are mutually influencing and promoting.

## Figures and Tables

**Table 1:** Definition of indicator variables of marine economy and marine cultural industry development.

Variable name	Indicators of marine economic development			Indicators of marine culture industry development		
	Gross ocean product (X1)	Total imports and exports (X2)	Total imports and exports (X2)	Disposable income of urban residents (X4)	Number of tertiary industry employees(X5)	Total number of books published (BP) (X6)
Variable abbreviation	GOP	MEV	FAI	UPDI	TIE	BP

Variable unit	100 million yuan	100 million dollars	100 million yuan	1 yuan	10000 people	10000 copies

Variable meaning	The development level of sea-related industries	Level of development of import and export trade	Level of infrastructure development	Living standards in marine areas	The employment level of people in maritime areas	The spiritual and cultural level of people in maritime areas

Variable source	China oceanic statistical yearbook China marine economic development report	Fujian statistical yearbook 2020	Fujian statistical yearbook 2020	Fujian statistical yearbook 2020	Fujian statistical yearbook 2020	Fujian statistical yearbook 2020

**Table 2:** The percentage of ocean culture industry ocean transportation and marine fishery.

Years	Marine culture industry	Transportation	Fisheries
2009	16.09	13.83	10.15
2010	19.31	13.37	9.68
2011	13.22	14.66	9.58
2012	14.83	13.85	8.67
2013	16.27	13.44	8.54
2014	17.33	11.72	7.74
2015	17.99	11.85	7.44
2016	18.11	11.78	7.5
2017	19.26	9.75	7.56
2018	19.14	9.57	7.21
2019	19.59	8.7	7.22
2020	19.89	9.59	7.29

**Table 3:** Ocean culture industry income elasticity of demand.

Year	Marine culture industry		Per capita GDP		Income elasticity of demand
	Output value (hundred million Rmb)	The growth rate (%)	GDP (RMB)	Appreciation (%)	
2012	2174.29	37.64	12336	17.02	2.21
2013	2872.29	32.1	14185	14.99	2.14
2014	3742.29	30.29	16500	16.32	1.86
2015	4608.29	23.14	20169	22.24	1.04
2016	5380.57	16.76	23708	17.55	0.96
2017	6217.57	15.56	25608	8.01	1.94
2018	7575.86	21.85	30015	17.21	1.27
2019	8914.14	17.67	35181	17.21	1.03
2020	9960	11.73	37195	5.72	2.05

**Table 4:** Ocean-Related employment elasticity.

Year	Number of sea-related jobs nationwide		Marine culture industry		Elasticity of employment
	People (10000)	Appreciation (%)	Production value	Appreciation (%)	
2015	2960.3	6.45	870	30.29	0.21
2016	3151.3	6.45	866	23.14	0.28
2017	3218.3	2.13	772.29	16.76	0.13
2018	3270.6	1.63	837	15.56	0.1
2019	3350.8	2.45	1358.2	21.85	0.11
2020	3421.2	2.1	1338.29	17.67	0.12

**Table 5:** Table of raw data.

Year	Indicators of marine economic development			Indicators of marine culture industry development		
	X1	X2	X3	X4	X5	X6
	GOP	MEV	FAI	UPDI	TIE	BP
1990	130.6	43.39	90.51	1749	284.34	16312
1991	154.9	57.48	117.28	1953	306.14	17667
1992	196.2	80.59	193.21	2351	324.92	19399
1993	278.6	100.42	320.45	2923	356.64	17044
1994	411.1	121.9	472.49	3935	386.67	19745
1995	523.7	144.46	594.45	4853	407.98	18448
1996	621.1	155.2	696.91	5574	424	21348
1997	717.7	179.53	794.33	6144	433.34	23282
1998	789.9	171.61	941.25	6486	445.56	21596
1999	853.5	176.2	952.22	6860	452.22	21875
2000	941.1	212.23	995.38	7432	476.71	20298
2001	1018.2	226.26	1053.84	8313	489.94	17891
2002	1116.9	283.99	1148.76	9189	499.58	19953
2003	1249.9	353.26	1411.45	10000	523.6	15595
2004	1428.0	475.27	1789.38	11175	551.55	13907
2005	1603.9	544.11	2241.70	12321	583.69	10643
2006	1867.1	626.59	2998.45	13753	616.43	9840
2007	2290.3	744.51	4186.67	15505	649.79	8463
2008	2688.2	848.21	5148.31	17961	692.24	7793
2009	3201.9	796.49	6180.94	19577	754.55	7689
2010	3682.9	1087.8	8067.33	21781	784.16	7749
2011	4284	1435.22	9885.67	24907	883.66	8294
2012	4482.8	1559.38	12452.24	28055	929.95	9078
2013	5028	1693.22	15245.24	28174	940.56	8870
2014	5980.2	1774.08	18141.37	30722	1021.04	8619
2015	7075.6	1688.46	21300.91	33275	1124.84	8800
2016	7999.7	1568.19	23107.49	36014	1175.39	9709
2017	8460.61	1710.35	26226.6	39001	1199.56	10809
2018	9671.9	1875.76	29400.1	42121	1224.15	11461
2019	10598.8	1930.86	31164.1	45620	1322.76	14385

**Table 6:** ADF unit root test results.

Variable	The ADF statistics	1% critical value	5% critical value	10% critical value	*P* value	Conclusion
GOP	−0.167666	−4.440739	−3.632896	−3.254671	0.9895	Nonstationary
1	−0.806893	−4.440739	−3.632896	−3.254671	0.9494	Nonstationary
2	−3.795812	−3.78803	−3.012363	−2.646119	0.0098	Stationary
MEV	−2.108362	−4.323979	−3.580623	−3.225334	0.5191	Nonstationary
1	−3.432349	−3.689194	−2.971853	−2.625121	0.0182	Stationary
2	−3.565382	−4.440739	−3.632896	−3.254671	0.0262	Nonstationary
FAI	−3.705701	−4.440739	−3.632896	−3.254671	0.0435	Stationary
1	−2.444314	−4.467895	−3.644963	−3.261452	0.3488	Nonstationary
2	−1.537274	−2.653401	−1.953858	−1.609571	0	Nonstationary
UPDI	1.085927	−4.309824	−3.574244	−3.221728	0.9998	Nonstationary
1	−4.656108	−4.323979	−3.580623	−3.225334	0.0046	Stationary
2	−5.227024	−4.374307	−3.603202	−3.238054	0.0015	Stationary
TIE	−3.644226	−4.416345	−3.622033	−3.248592	0.0479	Stationary
1	−4.961781	−4.33933	−3.587527	−3.22923	0.0024	Stationary
2	−5.270766	−3.737853	−2.991878	−2.635542	0.0003	Stationary
BP	−1.007396	−4.309824	−3.574244	−3.221728	0.9274	Nonstationary
1	−4.998777	−4.323979	−3.580623	−3.225334	0.0021	Stationary
2	−7.1565	−4.356068	−3.595026	−3.233456	0	Stationary

**Table 7:** Residual sequence equation.

*y* = −845.3336 + 0.230464 × 4 + *e*		*T* = (−5.715153) (32.85507)	
*R*-squared	0.974717	Durbin-Watson stat	0.211102
*y* = −3609.563 + 9.75216 × 5 + *e*		*T* = (−14.04658) (28.14606)	
*R*-squared	0.965862	Durbin-Watson stat	0.199081
*y* = 7854.884–0.342973 × 6 + *e*		*T* = (5.809431) (−3.840637)	
*R*-squared	0.345037	Durbin-Watson stat	0.112765

**Table 8:** Co-integration test table.

Variable	The ADF statistics	*P* value	1% critical value	5% critical value	10% critical value	Conclusion	Whether cointegration or not
*e*1	−0.745693	0.3783	−2.708094	−1.962813	−1.606129	Nonstationary	NO
*e*2	−2.153314	0.034	−2.717511	−1.964418	−1.605603	Stationary	YES
*e*3	−2.337891	0.0229	−2.717511	−1.964418	−1.605603	Stationary	YES

**Table 9:** Data table of the VAR model modeling.

	DDX1	DDX4	DDX5	DDX6
DDX1(− 1)	− 0.513044	2.132396	0.093531	3.942955
	− 0.29548	− 0.84005	− 0.02559	− 2.22456
	[− 1.73632]	[2.53842]	[3.65433]	[1.77246]
DDX1(− 2)	0.108172	3.281957	0.003807	3.648091
	− 0.57236	− 1.62723	− 0.04958	− 4.30913
	[0.18899]	[2.01689]	[0.07678]	[0.84660]
DDX4(− 1)	− 0.079658	− 0.505913	0.004796	1.127483
	−0.08635	− 0.24549	− 0.00748	− 0.65009
	[− 0.92251]	[− 2.06082]	[0.64126]	[1.73434]
DDX4(− 2)	− 0.064841	0.154699	− 0.009926	1.311395
	− 0.09473	− 0.26933	− 0.00821	− 0.71323
	[− 0.68445]	[0.57438]	[− 1.20955]	[1.83868]
DDX5(− 1)	− 0.900965	− 9.323938	− 0.863149	− 36.79936
	− 3.16212	−8.98995	− 0.27391	− 23.8066
	[− 0.28492]	[− 1.03715]	[− 3.15126]	[− 1.54577]
DDX5(− 2)	− 2.828118	− 25.25666	− 0.384216	− 27.77185
	− 3.68634	− 10.4803	− 0.31931	− 27.7533
	[− 0.76719]	[− 2.40991]	[−1.20325]	[− 1.00067]
DDX6(− 1)	− 0.004557	− 0.047359	− 0.001363	− 1.107571
	−0.02578	− 0.07331	− 0.00223	− 0.19412
	[− 0.17672]	[− 0.64605]	[− 0.61047]	[−5.70553]
DDX6(− 2)	− 0.007529	− 0.054228	− 0.000883	− 0.481722
	− 0.02635	− 0.0749	− 0.00228	− 0.19835
	[− 0.28576]	[− 0.72398]	[− 0.38698]	[− 2.42864]
C	69.22711	− 0.19971	− 0.977217	− 334.0393
	− 53.4736	− 152.026	− 4.63193	− 402.585
	[1.29460]	[0.00131]	[− 0.21097]	[− 0.82974]

**Table 10:** Table of lagging orders.

Lag	LogL	LR	FPE	AIC	SC	HQ
0	−694.6564	NA	2.27*E* + 20	58.22137	58.41771	58.27346
1	−661.899	51.86593^*∗*^	5.75*E* + 19	56.82492	57.80663	57.08537
2	−645.9779	19.90145	6.58*E* + 19	56.83149	58.59857	57.3003
3	−619.5644	24.21237	3.98*E* + 19	55.9637	58.51615	56.64086
4	−575.3092	25.81553	9.16*e* + 18^*∗*^	53.60910^*∗*^	56.94692^*∗*^	54.49462^*∗*^

**Table 11:** Granger causality test table.

Dependent variable: DDX1			
Excluded	Chi-sq	Df	Prob.
DDX4	11.47044	4	0.0218
DDX5	6.089166	4	0.1926
DDX6	2.708171	4	0.6078
All	47.38088	12	0

Dependent variable: DDX4			
Excluded	Chi-sq	Df	Prob.
DDX1	18.52228	4	0.001
DDX5	4.408588	4	0.3535
DDX6	3.751793	4	0.4406
All	42.26041	12	0

Dependent variable: DDX5			
Excluded	Chi-sq	Df	Prob.
DDX1	8.865778	4	0.0645
DDX4	8.656245	4	0.0703
DDX6	1.205154	4	0.8772
All	28.45182	12	0.0047

Dependent variable: DDX6			
Excluded	Chi-sq	Df	Prob.
DDX1	6.004358	4	0.0988
DDX4	1.468352	4	0.8322
DDX5	1.493952	4	0.8277
All	7.957921	12	0.7884

**Table 12:** Summary description of Granger causality test.

Explained variable	Explanatory variables	Granger causality test
GOP	UPDI	Accept
	TIE	Reject
	BP	Reject
UPDI	GOP	Accept
TIE	GOP	Accept
BP	GOP	Accept

## Data Availability

The experimental data used to support the findings of this study are available from the corresponding author upon request.

## References

[1] Charles S. C. (2003). *A Report of National Ocean Economics Project*.

[2] Rochwulaningsih Y., Sulistiyono S. T., Masruroh N. N., Maulany N. N. (2019). Marine policy basis of Indonesia as a maritime state: the importance of integrated economy. *Marine Policy*.

[3] Winther J. G., Dai M., Rist T. (2020). Integrated ocean management for a sustainable ocean economy. *Nature Ecology & Evolution*.

[4] Lubchenco J., Haugan P. M., Pangestu M. E. (2020). Five priorities for a sustainable ocean economy. *Nature*.

[5] Solow R. M. (1957). Technical change and the aggregate production function. *The Review of Economics and Statistics*.

[6] Lucas R. E. (1988). On the mechanics of economic development. *Journal of Monetary Economics*.

[7] Romer P. M. (1990). Endogenous technological change. *Journal of Political Economy*.

[8] Grossman G. M., Helpman E. (1991). Innovation and growth in the global economy.

[9] Grossman G. M., Helpman E. (1991). Quality ladders and product cycles. *Quarterly Journal of Economics*.

[10] Grossman G. M., Helpman E. (1991). Quality ladders in the theory of growth. *The Review of Economic Studies*.

[11] Acemoglu D. (2002). Directed technical change. *The Review of Economic Studies*.

[12] Dixit A. K., Stiglitz J. E. (1977). Monopolistic competition and optimum product diversity. *The American Economic Review*.

[13] Soug M., Wang S. (2018). Measuring environment-biased technological progress considering energy saving and emission reduction. *Process Safety and Environmental Protection*.

[14] Li J., See K. F., Chi J. (2019). Water resources and water pollution emissions in China’s industrial sector: a green-biased technological progress analysis. *Journal of Cleaner Production*.

[15] Wei Z., Han B., Han L., Shi Y. (2019). Factor substitution, diversified sources on biased technological progress and decomposition of energy intensity in China’s high-tech industry. *Journal of Cleaner Production*.

[16] Hicks J. R. (1963). *The Theory of Wages*.

[17] Maravelias C. D., Tsitsika E. V. (2008). Economic efficiency analysis and fleet capacity assessment in Mediterranean fisheries. *Fisheries Research*.

[18] Yu M. M., Hsu C. C. (2012). Service productivity and biased technological change of domestic airports in Taiwan. *International Journal of Sustainable Transportation*.

[19] Zheng H., Zhang J. C., Zhao X., Mu H. R. (2020). Exploring the affecting mechanism between environmental regulation and economic efficiency: new evidence from China’s coastal areas. *Ocean & Coastal Management*.

[20] Nadiri M. I. (1993). Innovations and technological spillovers. *Working Papers*.

[21] Chen J., Wang Y., Song M., Zhao R. (2017). Analyzing the decoupling relationship between marine economic growth and marine pollution in China. *Ocean Engineering*.

